The article "A COVID-19 Auxiliary Diagnosis Based on Federated Learning and Blockchain" was published in 2022. Journal: Comput Math Methods Med.

# A COVID-19 Auxiliary Diagnosis Based on Federated Learning and Blockchain

**DOI:** 10.1155/2022/7078764

**Published:** 2022-08-24

**Authors:** Ziyu Wang, Lei Cai, Xuewu Zhang, Chang Choi, Xin Su

**Affiliations:** ^1^College of IoT Engineering, Hohai University, Changzhou 213022, China; ^2^Department of Computer Engineering, Gachon University, Seongnam-si 13120, Republic of Korea

## Abstract

Due to the high transmission rate and high pathogenicity of the novel coronavirus (COVID-19), there is an urgent need for the diagnosis and treatment of outbreaks around the world. In order to diagnose quickly and accurately, an auxiliary diagnosis method is proposed for COVID-19 based on federated learning and blockchain, which can quickly and effectively enable collaborative model training among multiple medical institutions. It is beneficial to address data sharing difficulties and issues of privacy and security. This research mainly includes the following sectors: in order to address insufficient medical data and the data silos, this paper applies federated learning to COVID-19's medical diagnosis to achieve the transformation and refinement of big data values. With regard to third-party dependence, blockchain technology is introduced to protect sensitive information and safeguard the data rights of medical institutions. To ensure the model's validity and applicability, this paper simulates realistic situations based on a real COVID-19 dataset and analyses problems such as model iteration delays. Experimental results demonstrate that this method achieves a multiparty participation in training and a better data protection and would help medical personnel diagnose coronavirus disease more effectively.

## 1. Introduction

Epidemic novel coronavirus (COVID-19) [1] has being spreading since 2019, with high morbidity, transmission, and mortality rate. There is an urgent worldwide need for a prompt and accurate diagnosis, together with an effective treatment. Meanwhile, biomedical imaging has become an indispensable diagnosis tool in clinical trials [2, 3]. Currently, human-induced analysis to numerous images alone in medical institutions consumes a lot of human, material, and financial resources. Deep learning, as a forefront technology in the smart healthcare system, is bound to find a wide application in this field [4].

Implementing smart healthcare with traditional artificial intelligence approaches requires cloud servers or data centers to share local datasets. Such cloud servers have a computing power to provide efficient data training and analysis, whose abuse and malfunction may result in leakage of health information or compromise of sensitive data [5]. Even without authorization, attackers have a potential access to AI centers or third parties, such as the cloud server, for data. Similarly, they may control and modify data without a client's awareness or permission [6], while an efficient AI model inevitably needs numerous data to support training [7, 8]. Data exchanges among medical institutions partially support model training, but diversified institutional policies, privacy issues, and high costs hinder dataset sharing between institutions for model training purposes [9]. Against this background, current issues in smart healthcare manifest as how to achieve a secure sharing of medical data, overcoming data silos, and protecting sensitive private information.

Federated learning (FL), first put forward in 2016 [10], enables data sharing as well as model coconstruction without leaking respective data privacy. After that, smart healthcare undergoes rapid development in the federated learning ecosystem. Xu et al. [11] provide federated learning application scenarios in biomedicine and confirmed its feasibility in smart healthcare. In a federated learning-based healthcare system, AI only needs to train local models to upload parameters, while a central server updates the global picture, thus reducing the sensitive information leakage risk [12, 13]. Being immutable and traceable [14], blockchain is an effective tool to help decentralize federated learning. Timely updates of local model parameters are uploaded by clients to the blockchain's distributed ledgers, and these model updates are audited. All transaction records are tamper-evident and repudiation-resistant, with or without an authoritative inspection. In addition, differences in communicating and computing power of client devices cause model iteration delays [15, 16]. Blockchain helps trace back and correlate with individual participants, analyze block generation times, data block propagation times, and forking rates. Blockchain applied in the healthcare sector also enables timely electronic healthcare data processing. It protects sensitive patient information privacy and ensures secure data sharing among multiple organizations. Federated learning and blockchain jointly applied in the novel coronavirus diagnosis are likely to achieve a globally secure epidemic data sharing without sensitive information leakage, significantly contributing to epidemic control together with life and property safeguarding [17].

At present, the bottleneck concerning intelligent healthcare lies in the collection of multiple global datasets with diverse features, which are inherently difficult to integrate [18]. Healthcare organizations are also highly sensitive to data privacy and security. It becomes a sharp issue to guarantee large-scale model training accuracy and secure data use. This paper accordingly designs a new federated learning (FL) and Blockchain-Based COVID-19 Auxiliary Diagnostic Model (FB-COVID-19 AD) with the following research details and innovations.

1. Federated learning is applied to COVID-19 diagnosis and partially breaks the bottleneck of low model performance due to insufficient medical data. The framework proposed here allows medical staff to reap the benefits of the feature learning without privacy worries
2. In response to federated learning's reliance on third parties, a blockchain-distributed ledger is introduced to protect sensitive information. Moreover, a public chain is adopted to ensure users' rights and interests, and the proof of work mechanism (PoW) is adopted for transaction consensus. At the same time, the model iteration delay is analyzed, and blockchain forking is taken into account to maintain model performance stability
3. Based on real datasets to simulate actual situations, an independently and identically distributed (IID) experiment and nonindependently and nonidentically distributed (non-IID) experiment are designed in this paper. It verifies the system model's effectiveness and applicability. Private data from multiple medical institutions are soundly available and invisible in the training process, with the training efficiency significantly improved

The remaining paper follows this structure.  Section 2 presents and compares relevant medical works in terms of federated learning and other technologies.  Section 3 introduces the FB-COVID-19 AD model and algorithms for the system operation in detail. Its effectiveness and applicability are compared and analyzed with other research results in Section 4.  Section 5 summarizes the paper.

## 2. Related Works

### 2.1. Federated Learning-Related Medical Image Researches

The healthcare industry has been profoundly undergoing a digital transformation based on artificial intelligence and big data. It triggers higher requirements for healthcare data collection and sharing. With information silos being a primary challenge for smart healthcare, secure data sharing becomes a real challenge as they are from worldwide hospitals and other medical institutions. Federated learning shows some promise for smart healthcare [19]. As multiple hospitals store their datasets locally, the model's updated parameters uploaded to the central server alone complete a global model update [20].

Federated learning expands dataset sources and results in a significant improvement in medical data training quality. A horizontal federated learning (HFL) on medical images confirms the framework's outperformance over individually trained models by 6.3% on average [21]. A vertical federated learning (VFL) combined with deep learning used external data to validate the model's generalization ability [22]. So, federated learning is liable for medical image processing. Data privacy issues are tackled with a federated learning framework to address and verify its good performance on different neural network classification models [23]. However, a federated learning framework alone is adopted as a solution to data sharing and data security here. Attention is not attached to the protection of model parameters in federated learning yet. Given the sensitivity and privacy of healthcare data, this model alone fails to meet current and immediate needs. Huge system losses are also possible if an attacker abuses model parameters to derive data.

Privacy data from medical institutions may also get leaked through the gradient information. Similarly, label and membership information may be launched by an attacker while issuing the uploaded model parameters. Differential privacy techniques are commonly applied to federated learning with regard to various privacy securities at the user's end. Federated learning on medical devices and differential privacy techniques (DP) in the system are adopted to protect information during model exchanges [24]. On this basis, a trade-off between privacy cost and model accuracy is implemented with Gaussian noise [25]. A Chinese study applies model parameters with Gaussian noise on the server side and adopts an adaptive gradient cropping strategy to enhance model performance [26]. A multisource diffusion image dataset accounts for variation between clients [27]. Each medical institution in these studies employs a generative adversarial network (GAN) to transform the original images into the target space to address the cross-client privacy protection. These articles all deal with data privacy protection through federated learning models and break data barriers between different medical institutions. Some consider algorithm optimization with differential privacy techniques to achieve either client-side or server-side data protection. Unfortunately, the central server itself remains untouched once it fails or gets paralyzed by attacks. The overall system model optimization also lacks, unable to ensure a system model's optimal performance.

### 2.2. Blockchain Involved Medical Image Researches

Section 2.1 discusses federated learning used to enable multiple parties to share data, only which it has to address dependency on third parties. Blockchain, as the underlying technology of Bitcoin, is essentially a decentralized database [28, 29]. Also, it is a technical solution to collectively maintain a reliable database using decentralization and detrust. Blockchain has brought together new technologies such as cryptography, distributed storage, smart contracts, and consensus algorithms. Blockchain combined in the healthcare sector is in line with the technological needs to support complex application scenarios [30]. The use of blockchain in a distributed federated learning healthcare system has already been studied to beat untrustworthy servers and external attacks, coordinating global model update computations in a peer-to-peer manner through institutions' block consensus [31].

Concerns in healthcare data mainly point to patient information sensitivity and dataset finiteness [32]. Blockchain has essential characteristics like “decentralization,” immutability, and anonymity, which effectively make up for the gap that federated learning relies on central nodes. In the long run, combining federated learning and blockchain helps artificial intelligence to develop in the medical field. Consortium chain and block authorization methods are used in federated learning, where each institution uses the local COVID-19 dataset to train the model and only uploads model parameters such as gradient updates [33]. In this method, a miner's failure to complete learning affects its connected clients in the blockchain. To deal with the issue, the miner unites other miners' clients to confirm the transaction [34]. In addition, a reputation value calculation method based on dual subjective logic is used in client screening to incentivize clients to participate in training [35].

Concentrating information on one server potentially brings about potential risks like attacks and unfairness to the system. As an indispensable tool for doctors' diagnosis, medical images have high data privacy protection requirements. In view of these, federated learning and blockchain combined well to meet diagnosis needs with medical images [36]. FL opens new opportunities for smart healthcare, but relevant literature is insufficient in terms of the system model latency and block forking, etc. Besides an adverse impact on the transaction confirmation time, they also have negative impacts on the system stability and global model accuracy.

This paper summarizes system solutions in medical imaging utilizing the federated learning framework, as shown in Table 1. A comprehensive comparison of existing medical diagnostic researches based on federated learning is presented in terms of technological coordination, client side, aggregation side, and application scope, respectively.

As summarized in Table 1, most healthcare systems use horizontal federated learning as the model framework to combine multiple medical institutions with the same characteristics for multisample learning. Most system models in the literature use common medical image datasets to evaluate the training effect and hopefully improve farsighted FL healthcare systems. Besides, regarding data privacy protection, some researches compensate for the shortcomings of FL in sensitive data protection by combining differentiated privacy protection and blockchain technology, etc. In brief, FL combined with other technologies is a very effective learning approach to accelerate the AI model training accuracy rates.

## 3. Materials and Methods

### 3.1. FB-COVID-19 AD Model

#### 3.1.1. Introduction

As shown in Figure 1, FB-COVID-19 AD sets multiple medical institutions as the client, the blockchain composed of public chains as the server. Apart from that, data exchanges between the client and the server are realized at an access node layer. Different medical institutions are successfully united to train the pneumonia image classification model. Each component is described in detail as follows:

1. Medical client layer: any owner of local medical image datasets. Based on the local dataset, each client trains models and uploads model parameters. At the same time, clients in this layer also accept global update parameters to export global model updates
2. Access node layer: a communication infrastructure with computing power. It receives model parameters uploaded by individual medical institutions, as well as downlinks block information from the blockchain service layer
3. Blockchain service layer: a complete transaction data owner and verifier. Using distributed data storage, several complete transaction data sets are stored in each block, and parameters are authenticated using consensus protocols

#### 3.1.2. Training in Medical Institutions

In FB-COVID-19 AD, since multiple medical institutions jointly participate in model training, they only need to provide model parameters to data requestors. Given the practicalities, data_*n*,*i*_ = {*x*_*n*,*i*_, *y*_*n*,*i*_} is the local dataset belonging to each medical institution, where *x*_*n*,*i*_ is the input sample vector of the *n*th hospital added to the current federated training. Similarly, *y*_*n*,*i*_ is its corresponding label vector. Data = ∑_*n*∈*N*_∑_*i*∈*I*_data_*n*,*i*_ is the total dataset participating in the current federated training, where *i* ∈ *I* denotes sample *i*, *n* ∈ *N* denotes medical institution *n*, and *N* denotes the set of all medical institutions. At the same time, *W*_*n*_ is the model parameters of the *n*th medical institution participating in the local training, and the local model update is uploaded to the blockchain node miner *M*_*t*_. Likewise, the set of input samples and the corresponding set of tags are set to *X*_*n*_, *Y*_*n*_. In the model training process, *F*_*n*_ is the objective function of the *n*th medical institution, and *f*_*n*_(*w*) is the corresponding local loss function, which is defined as follows:

(1) $$\begin{array}{c} F_{n}≜\min\left\{\frac{1}{N}\cdot \underset{n\in N}{\sum }f_{n}\left(w\right)\right\}. \end{array}$$

Using optimizers to find optimal values help solve the above equation minimization and improve model accuracy. In a traditional FL setup, it is the local updates that are uploaded to the federated server. For the FB-COVID-19 AD system model, it is the updates that are saved in the candidate blocks to be mined. Setting the learning rate to *e*, the model parameters for the *t*th iteration update in the *k*th round of the healthcare facility *n* are formulated as

(2) $$\begin{array}{c} w_{n}^{t,k}=w_{n}^{t-1,k}-e\cdot \nabla f\left(w_{n}^{k-1},x_{n,i},y_{n,i}\right). \end{array}$$

At the same time, the *k* round updated global weights are formulated as

(3) $$\begin{array}{c} w^{k}=\frac{1}{N}\cdot \overset{N}{\underset{n=1}{\sum }}\overset{I}{\underset{i=1}{\sum }}\frac{w_{n}^{k}\cdot {\text{data}}_{n}}{\text{Data}},\\ \nabla f\left(w^{k}\right)=\frac{1}{N}\cdot \overset{N}{\underset{n=1}{\sum }}\overset{I}{\underset{i=1}{\sum }}\nabla f\left(w_{n}^{k},x_{n},y_{n}\right). \end{array}$$

The updated local model gradient parameter {*w*_*n*_^*k*^, ∇*f*(*w*^*k*^)} is then uploaded to the server-side blockchain. The federated averaging algorithm (FedAvg) [9] is used to compute the global model gradient. When a new block is generated, the medical institution downloads the data about the new block from the miner and uses its aggregated results to compute *w*^*k*^ to update the model. In FL setup, the medical institution iterates the process until it satisfies the inequality: |*f*(*w*^*k*^) − *f*(*w*^*k*−1^)| ≤ *δ*, where *δ* ∈ *R* is the loss of precision.

#### 3.1.3. Blockchain Aggregation

By using the value representation and transfer function from blockchain, the value created by a local medical institution is tagged while the benefits are distributed. Each medical institution has its corresponding miners, all of whom are used as nodes to form the blockchain. The device uploads updated model parameters {*w*_*n*_^*k*^, ∇*f*(*w*^*k*^)} and the computing time used *T*_local,*n*_^*k*^ to its corresponding miners. To prevent unauthorized block copying, miners store the defined data structure Merkle trees and create new blocks at specific times, which contain unique hash values, block generation rate *λ*, Nonce values, timestamps, etc. To achieve a consistent state of the chain, all miners apply the consensus protocol PoW to implement mining to verify the new blocks. When mining is complete, the verified blocks are placed in candidate blocks and broadcast across the network. At this moment, parameters in the local model update are safely stored in the blockchain. The information from those accepted blocks is then used to derive the parameters of the global model update {*w*^*k*^, ∇*f*(*w*^*k*^)} for calculation. Clients in the model exchange local information via the blockchain, which keeps track of individual model updates and does not implement model aggregation via third parties. Through decentralized learning, the global model is constructed by local medical institutions or miners with sufficient computational power. The global model calculation is completed with individual medical institutions in this paper.

The consensus mechanism is the blockchain's core technology. It allows transactions to be conducted safely and reliably in a centralized network [37]. A public chain is used to achieve complete decentralization, and PoW is used as the consensus protocol to achieve distribution in correspondence to its workload. Miners compete for arithmetic power, constantly searching for the random number Nonce through their own arithmetic power [38]. Only the licensed miner has the right for bookkeeping, who first finds the Nonce value and broadcasts it to the whole network for recognition. The packaged candidate block is broadcasted to the network as a new block. Then, other miners stop computing and add the new block to the local ledger once they receive the message.

PoW provides a high degree of decentralization and robustness for large-scale blockchain. But in the process, different nodes tend to have different perspectives towards the blockchain due to differences in their arrival times. Hence, the process is termed as “Fork” (Figure 2). A chain fork may cause some clients to receive incorrect global model updates. Inevitably, it brings a negative effect to the next round of local model updates. Assuming that all miners work in parallel, the probability of the fork is defined as

(4) $$\begin{array}{c} p_{f}=1-e^{-\lambda \left(M-1\right)\beta_{BP}}, \end{array}$$

where *λ* is the block generation rate and 1/*λ* is the expected time for a block generation. Besides, *M* is the number of miners, and *β*_*BP*_ is the block body propagation delay. So, the block mining time is expressed as a Poisson process.

In the FB-COVID-19 AD process, the server-side blockchain provides a credible incentive for contribution to encourage more medical institutions to join and improve the data processing accuracy. All medical institutions are timely rewarded with a reference to their data quantity and quality. Simultaneously, miners *M*_*t*_ are rewarded according to the quantity and quality of data_*n*,*i*_ from the local medical institutions they are associated with. By writing the reward resources into the blockchain, the blockchain openness and transparency will attract more clients to join and improve the collaboration efficiency among medical institutions.

### 3.2. FB-COVID-19 AD Algorithm

#### 3.2.1. FB-COVID-19 AD Single Iteration Process

As shown in Figure 1, decentralization is realized through federated learning and blockchain combination. In FB-COVID-19 AD, FL clients' devices interact with the local model update parameters through the blockchain to achieve model aggregation without a third-party server. A single iteration of the local healthcare facility is implemented applying the following steps.

Local calculation: using the local dataset data_*n*,*i*_, each medical institution calculates *w*_*n*_^*k*^ through a local optimization mechanism.

Data upload: a miner is randomly connected to medical facilities which uploads the calculated parameters {*w*_*n*_^*k*^, ∇*f*(*w*^*k*^)} and time *T*_local,*n*_^*k*^ to the corresponding miner *M*_*t*_.

Block generation: while waiting for enough transactions to be received (determined by the maximum block size) or exceeding the maximum waiting time *τ*, a candidate block is generated for mining.

Block mining: with the consensus mechanism PoW, a random number Nonce is calculated to determine the next block to be added to the blockchain, or to receive a block broadcast by another miner.

Block propagation: *M*_*i*_ ∈ *M* is the first miner to complete the calculation. Propagate *M*_*i*_ the candidate block upload message through the P2P network.

Block download: the medical institution downloads the latest block via the corresponding miner *M*_*t*_.

Global model aggregation: local medical institutions use the information in the accepted blocks (local model updates) to calculate and derive global model updates.

The above operation steps continue until inequality |*f*(*w*^*k*^) − *f*(*w*^*k*−1^)| ≤ *δ* is satisfied. In step 7 of the above iteration, a global model update is done by the client, based on the differences in the miners' computing power. In fact, a failure is liable to affect the global model's update. For the IID dataset, the global model is initially downloaded by each medical institution itself and then updated using local data. Once the local model is updated, values of the model update parameters are uploaded to the blockchain to generate a new block to mine. The latest block will contain the global model parameters updated using all the local update parameters, so the block size is adapted to fit all update values. For the non-IID dataset, the medical institution submits the model update parameter values asynchronously after completing the local model update. A new block is generated when enough transactions have been received or when the maximum wait time *τ* has been exceeded. The specific algorithms for the FD-COVID-19 AD system model for the IID dataset and the non-IID dataset are shown in Algorithm 1 and Algorithm 2.

In the above steps, a block generation is determined by block size *S*_*B*_ and waiting time *τ*. Block size *S*_*B*_ is an important parameter in FB-COVID-19 AD. The larger the block size, the higher the information quality provided by a single iteration in federated learning, but the higher the fork rate and iteration latency time. Setting the block size correctly will affect the blockchain throughput and thus the completion time of federated learning. Block size optimization does not fall within the focus of this paper and is ignored for the time being.

#### 3.2.2. FB-COVID-19 AD Iterative Latency Analysis

Due to equipment performance differences, the network, and other factors, this section will focus on analyzing the running time of the FB-COVID-19 AD single iteration process in Section 3.2.1 and defining following delay time parameters:

1. Block fill delay *β*_*BF*_: a block is filled with data from step 2 to upload the local update. This contains the local model computation time (i.e., the time it takes for the client to update the local model gradient). Also, this includes the local model upload time (i.e., the time it takes for the client to hand over the model to the miner)
2. Block generation delay *β*_*BG*_: the time miners spend looking up random values of Nonce, or waiting to receive a new valid block, as calculated by the PoW consensus mechanism
3. Block propagation delay *β*_*BP*_: the full network propagation of the mined blocks is achieved through a P2P network, assuming that all miners receive the propagated blocks at the same time
4. Global model aggregation delay *β*_*AG*_: the block downloading process in step 6 is executed first, and then, the client aggregates the local model information from the newly mined blocks to calculate the global model update
5. Block download latency *β*_*BD*_: the client downloads the latest block propagated from the miner, which contains either the local model updated in the last iteration or the global model. It depends on the model aggregation method

By calculating all delay times in the FB-COVID-19 AD process, and by considering the effect of bifurcation *p*_*f*_, the expected iteration delay time was defined as:

(5) $$\begin{array}{c} T_{\text{iter}}^{k}=\frac{\left(\beta_{BF}+\beta_{BG}+\beta_{BP}\right)}{1-p_{f}}+\beta_{AG}+\beta_{BD}. \end{array}$$

As block filling, block generation, and block propagation are all affected by the fork, these steps will be repeated once a conflict occurs.

## 4. Results and Discussion

### 4.1. The Dataset and Evaluating Indicators

A CT map dataset of COVID-19 is used (Figure 3) from the reference [39], created by collating from several public databases as well as recently published articles. A typical COVID-19 patient's chest image appears white on CT, and the shade depth correlates to its lesion gravity. At an earlier stage of the symptom, there may be multiple small patchy shadows as well as interstitial changes. Then, it would develop into multiple ground-glass shadows, infiltrative shadows, and lung consolidation in severe cases [3]. Accordingly, this dataset is filtered which contains 1313 CT maps of normal chests, 1316 CT maps of novel coronavirus diseases and 1171 CT maps of COVID-19 diseases. The entire dataset is divided into a training set, a test set, and a validation set. Accordingly, the basic information on the division of the dataset is shown in Table 2.

In this paper, the accuracy ACC is set as the evaluation index. The larger the ACC value, the higher the accuracy of the model's classification. As long as the samples are correctly predicted, the formula numerator will automatically increase by one, and the denominator will still represent all samples.

(6) $$\begin{array}{c} \text{ACC}=\frac{{\text{TP}}_{n}+\text{T}{\text{N}}_{n}}{{\text{TP}}_{n}+\text{F}{\text{P}}_{n}+\text{F}{\text{N}}_{n}+\text{T}{\text{N}}_{n}}, \end{array}$$

where TP_*n*_, TN_*n*_, FP_*n*_, and FN_*n*_ represent true positive, true negative, false positive, and false negative for the corresponding healthcare facility clients, respectively, where *n* is the *n*th hospital. The confusion matrix is shown in Table 3.

### 4.2. Numerical Results and Discussion

The information about the implementation of our software and hardware platforms is shown in Table 4. The local medical institution uses residual networks to train model. Some training hyperparameters were set as: the initial learning rate is 0.005, momentum is 0.5, and a ReLu function serves as the activation function. To ensure the comparison accuracy of experimental results, the time for each block generation in the model blockchain should remain as consistent as possible with the time for the parameter aggregation using the central server in FL based on FedAvg.

To verify the effectiveness of FL to address the data silos, an experiment of training 20 clients with different sized IID samples is conducted. As is shown in Figure 4, we compare the classification accuracy of the proposed model using all distributed samples with the best model and the worst model of the local training clients. It is apparent that the model obtained from the joint multiparty participation training is better than the one trained by medical institutions alone. In terms of accuracy, the model training accuracy in this paper has a 1.01% margin higher than that of the medical institution with the best training effect on average. At the same time, the model training enjoys a 4.61% effectiveness margin on average in this paper over that of the worst institution's training effectiveness. It soundly confirms multiparty participation training with apparent improvements of the model training effect.

As is shown in Figure 5, an experiment is conducted to compare the centralized training model, the proposed model, and the FL model. Clients of FL models upload model parameters through parallel training and carry out aggregated computation through the FedAvg algorithm. It is clear that a blockchain introduction to FL for decentralization does not cause a negative impact on the classification performance from these accuracy curves.

In a practical scenario, samples of the dataset are distributed at different medical institutions with distinct quality, quantity, and nonindependent identically distribution. The difference in the training samples makes it difficult to ensure that the model update operation is consistent for each participant. In Table 5, centralized training using all samples has higher accuracy than both the proposed and FL model based on FedAvg using distributed samples. However, there is a potential for the asynchronous method in the FL process since it achieves similar performance when using non-IID datasets.

Due to PoW operation, the performance of the FB-COVID-19 AD model can be hindered by forks. The fork splits the BC into different states and potentially undermines the overall agreement between participants. In the experiment, different numbers of miners are set as *M* = {10, 100, 500}, and consider different link capacities Cap = {1Mps, 5Mps, 20Mps}. As is shown in Figure 6, the fork rate increases with the number of federated learning participants, which requires a change in the block size to contain more parallel transactions. At the same time, with the same number of miners, the fork rate decreases as the link capacity increases. This phenomenon becomes more pronounced when the number of miners *M* = 100 and *M* = 500, respectively. These results confirm that in larger model networks, the link capacity needs to be increased for the exchange between miners to reduce the fork rate. Thus, it helps to reduce exchange time during the process.

The relationship between iteration delay time *T*_iter_, fork rate *p*_*f*_, and block generation rate *λ* was analyzed for different link capacities. As is shown in Figure 7, Cap = {1Mps, 20Mps, 50Mps} have three cases with different link capacities. In these cases, the fork rate is rising with the block generation rate increase. Meanwhile, the iteration delay time decreases, and the trend manifests a concave shape. The comparison of the three link capacities illustrates that the link capacity increase leads to a reduced impact of the fork rate. The iteration delay time decreases as the link capacity increases.

## 5. Conclusion

This paper mainly designs a method for auxiliary COVID-19 diagnosis through a combination of federated learning and blockchain technologies. Federated learning is used to address data barriers as well as insecure data sharing. Blockchain achieves decentralization, protects medically sensitive information, and encourages more medical institutions to participate in collaborative training. The proposed method is tested on a COVID-19 image dataset and achieves the expected training results. Compared with the centralized training, FB-COVID-19 AD model achieves collaborative cooperation among multiple participants without significant sacrifice of diagnostic accuracy. At the same time, experiments also investigate the single iteration latency of the system model and analyze the relationship between parameters such as fork rate, number of miners, block generation rate, and block capacity. In the future of smart healthcare, federated learning combined with other privacy and security technologies such as blockchain and differential privacy are expected to provide more innovative ideas for a secure sharing of healthcare data. Amidst the current global epidemic situations, federated learning and blockchain combined points to an important breakthrough for algorithmic models designed to assist epidemic diagnosis.

## Figures and Tables

**Figure 1:** FB-COVID-19 AD.

**Figure 2:** Blockchain fork.

**Figure 3:** Images in the dataset.

**Figure 4:** Differences in training accuracy of medical institutions.

**Figure 5:** Three methods to train curves.

**Figure 6:** Fork rate versus number of clients and number of miners.

**Figure 7:** Delay time versus fork rate and block generation rate.

**Algorithm 1:** FB-COVID-19 AD (IID).

**Algorithm 2:** : FB-COVID-19 AD (non-IID).

**Table 1:** Comparison of healthcare systems programs based on federated learning.

Ref.	FL type	Technology	Clients	Aggregator	Dataset type	Application
[19]	HFL	/	Hospital	Data center	Acute neurological disorders	Object detection
[21]	HFL	/	Medical sites	Federated sever	Breast density classification	Image classification
[22]	VFL	/	Hospital	Federated sever	COVID-19	Object detection
[23]	HFL	/	Hospital	Federated sever	Pneumonia	Image classification
[24]	HFL	DP	MRI machines	Federated sever	Brain tumour	Image segmentation
[25]	HFL	DP	Hospital	Data center	Diabetic retinopathy	Image classification
[26]	HFL	DP	Medical sites	Federated sever	Multitype lesion map	Object detection
[27]	VFL	GAN	Hospital	Cloud sever	Prostate cancer	Image classification
[31]	VFL/HFL	Blockchain	Smart service	Blockchain	/	/
[33]	HFL	Blockchain	Hospital	Blockchain	COVID-19	Image segmentation/class
[34]	HFL	Blockchain	Medical sites	Blockchain	COVID-19	Image segmentation
[35]	HFL	Blockchain	Hospital	Blockchain	MNIST	Image classification

**Table 2:** Dataset distribution.

	Normal	Viral	COVID-19	Total
Train	1113	1116	971	3200
Test	180	180	180	540
Valid	20	20	20	60

**Table 3:** Confusion matrix.

Prediction Labe	Real label	
	Positive	Negative
Positive	True positive	False positive
Negative	False negative	True negative

**Table 4:** Software and hardware environments.

Term	Total
CPU	INTEL I9-12900K
GPU	NVIDIA RTX3090
Video memory	48 G
Internal memory	128 G
Operating system	Ubuntu 20.04
Development language	Python 3.7

**Table 5:** The accuracy of three methods on COVID-19 dataset.

Method	Centralized training	FB-COVID-19 AD IID	FL-FedAvg IID	FB-COVID-19 AD non-IID	FL-FedAvg non-IID
Epoch = 20	0.901	0.903	0.881	0.728	0.738
Epoch = 40	0.931	0.923	0.892	0.847	0.835
Epoch = 60	0.960	0.931	0.923	0.917	0.903
Epoch = 80	0.946	0.933	0.929	0.932	0.923
Epoch = 100	0.963	0.947	0.940	0.933	0.923

## Data Availability

The data used to support the findings of this study are available from the corresponding author upon request.
